# Histopathological Analysis of Central Nervous System Metastases: Six Years of Data From a Tertiary Center

**DOI:** 10.7759/cureus.22151

**Published:** 2022-02-12

**Authors:** Zeynel Abidin Tas, Ozgur Kulahci

**Affiliations:** 1 Pathology, Health Sciences University Adana City Training and Research Hospital, Adana, TUR

**Keywords:** immunohistochemistry, histology, incidence, metastasis, central nervous system

## Abstract

Introduction: The most common cause of neurological symptoms in patients with systemic malignant tumors is central nervous system (CNS) metastases, and CNS metastases are one of the important causes of morbidity and mortality in these patients. The most common metastatic tumors to the CNS are lung, breast, malignant melanoma, genitourinary, and gastrointestinal tumors. We aimed to analyze our data on patients with CNS metastases in our department, which belongs to a large archive in the field of neuropathology.

Methods: The data of patients who had CNS metastases between January 2015 and August 2021 in our department were reviewed retrospectively. The patients were grouped in terms of demographic data, location, histopathological diagnosis, and primary origin characteristics, and their frequency and immunohistochemical staining characteristics were investigated.

Results: There were 256 patients with CNS metastases in our study. The mean age was found to be 56.12. Of the patients, 30.5% were female and 69.5% were male. Astrocytic and oligodendral tumors (25.3%), followed by meningiomas (24.1%), and then CNS metastases (21.3%) were the most common CNS tumors. Among the CNS metastases, the most common primary sites were the lung (58%), breast (16%), tumors of unknown primary origin (TUP) (5%), colon (4%), and gynecologic tract (3.1%). Localization was found as cerebral (69.5%), cerebellar (28.1%), and spinal (2.3%).

Conclusion: In CNS system metastases, an accurate histological diagnosis should be made by histomorphological evaluation supported by compatible immunohistochemical results in the presence of clinical history and radiological findings. Despite performing a larger immunohistochemical panel, it should be kept in mind that a primary site of origin cannot be found in a significant number of cases.

## Introduction

The WHO classification of central nervous system (CNS) tumors is subdivided into primary and metastatic tumors. While diagnostically confirmed or unconfirmed primary CNS tumors constitute 85%-90% of all brain tumors, metastatic tumors are seen in approximately 10%. Brain metastases were found in 25% of patients who died of cancer in autopsy studies [1,2]. Metastases are less common in the pediatric age group and more common in adults [1]. Brain metastases most commonly arise from tumors of the gastrointestinal system (GIS), prostate, and lung in men and tumors of the breast, GIS, and gynecologic tract in women. Likewise, the most common histological type varies according to the age of the patient. The most common cancer that metastasizes to the brain in adults is lung cancer, especially adenocarcinoma and small cell lung carcinoma [1,3]. These are followed by breast cancer, malignant melanoma, renal cell carcinoma, and colorectal carcinoma. Prostate, breast, and lung cancers are the most common cancers with spinal/epidural metastases. Head and neck tumors can metastasize to the CNS by direct spread. The most common cancers that metastasize to the brain in childhood are leukemia and lymphomas, followed by germ cell tumors, osteosarcoma, neuroblastoma, Ewing sarcoma, and rhabdomyosarcoma. CNS metastases are seen 80% in the cerebral hemispheres, 15% in the cerebellum, and 5% in other areas of the CNS. CNS metastases, which mostly manifest with symptoms of increased intracranial pressure in the clinic, may present in some patients as intracranial hemorrhage and infarction areas that can be easily recognized by magnetic resonance imaging (MRI) and computed tomography (CT). CNS metastases are often described macroscopically as round-oval-shaped, gray-white, or flesh-colored masses with or without central necrosis in the brain and spinal cord. It can be solitary or multifocal. Sometimes, changes similar to the features of the primary tumor, such as mucoid material in adenocarcinoma metastases, can also be seen. The histological and immunohistochemical features of CNS metastases are similar to those of the primary tumor from which they originate. Most metastases exhibit a fairly well-circumscribed, perivascular growth pattern, while small cell carcinomas and lymphomas may show infiltrative growth [1,4,5].

Immunohistochemical workup provides a valuable aid in the differentiation of primary and secondary tumors. Immunohistochemical markers (cytokeratin (CK) 5/6, cluster of differentiation 56 (CD56), CK7, CK20, thyroid transcription factor 1 (TTF-1), napsin A, GCDFP-15, caudal type homeobox transcription factor 2 (CDX2), RCC, PSA, EMA, PAX8, vimentin, melanoma antigen (Melan-A), leukocyte common antigen (LCA), chromogranin, synaptophysin, SOX10, and p63) that are frequently used in the approach to CNS metastases, except in exceptional cases, are very useful for the diagnosis of the primary tumor [6].

We aimed to present the data of our department, where many cases were diagnosed in the field of neuropathology, and to compare them with the literature.

## Materials and methods

We retrospectively analyzed the data of patients aged 3-90 years who were operated on for CNS mass in Adana City Training and Research Hospital between January 2015 and August 2021 and were diagnosed with CNS metastasis. Nonneoplastic central nervous system lesions were excluded from the study. Approval was obtained from Health Sciences University Adana City Training and Research Hospital Ethics Committee (approval number: 1591). The hematoxylin and eosin-stained sections of formalin-fixed paraffin-embedded tissues were evaluated. In addition to histopathological evaluation, glial fibrillary acidic protein (GFAP), pan-cytokeratin (PanCK), cytokeratin 7 (CK7), cytokeratin 20 (CK20), thyroid transcription factor 1 (TTF-1), synaptophysin, chromogranin, cluster of differentiation 56 (CD56), caudal type homeobox transcription factor 2 (CDX2), melanoma antigen (Melan-A), p63, p40, estrogen receptor (ER), and GATA3 staining results used for different cases were reviewed. GFAP and epithelial markers (cytokeratins) were used in those tumors where the differential diagnoses were between primary tumors of glial origin and metastases. Markers such as synaptophysin, chromogranin, and CD56 were used to demonstrate neuroendocrine differentiation. LCA was used to exclude tumors of lymphoid origin. Melan-A, GATA3, ER, and TTF-1 were used to confirm the diagnosis of specific tumors. Immunohistochemistry (IHC) was done on three-micron paraffin sections on 3‑aminopropyltriethoxysilane-coated slides, using prediluted antibodies, with known positive controls by polymer horseradish peroxidase (HRP) IHC detection system, following the manufacturer’s instructions. The slides were stained with 3, 3′‑diaminobenzidine tetrahydrochloride (DAB) chromogen, counterstained with hematoxylin, and mounted. The GATA3 antibody was from Cell Marque (Rocklin, CA, USA), and the p40 antibody was from Zeta Corporation (Sierra Madre, CA, USA). All the other antibodies were from Leica (Wetzlar, Germany). We analyzed the distribution of patients in terms of age, gender, location, and primary origin. Age was entered in years. Gender was grouped as male and female. Localization was grouped as cerebral, cerebellar, and spinal. The SPSS 19 package program was used for the statistical evaluation of the data obtained in the study (IBM Corporation, Armonk, NY, USA). The continuous variable was summarized as mean age. Gender, location, and categorical variables such as primary origin and histological type were summarized as numbers (n) and percentages (%).

## Results

There were 256 patients with CNS metastases in our study. The ages of the patients ranged from three to 90 years. The mean age was found to be 56.12. Of the patients, 30.5% were female and 69.5% were male. Among all central nervous system tumors, astrocytic and oligodendral tumors were 25.3%, meningiomas were 24.3%, and metastatic tumors were 21.3%. While the mean age was 48.82 among all central nervous system tumors, it was 53.15 in astrocytic and oligodendral tumors, 55.78 in meningiomas, and 56.12 in metastatic tumors. The proportional distribution of CNS tumors is summarized in Table 1.

**Table 1:** Age and gender characteristics of patients with central nervous system tumors

	n (%)	Female (n (%))	Male (n (%))	Mean age (years)
Astrocytic and oligodendral tumors	305 (25.3)	121 (39.7)	184 (60.3)	53.15
Other astrocytic tumors	34 (2.8)	18 (53)	16 (47)	17.11
Ependymal tumors	43 (3.6)	14 (32.6)	29 (67.4)	36.04
Choroid plexus tumors	8 (0.7)	3 (37.5)	5 (62.5)	38.50
Neuronal and glioneuronal tumors	12 (1)	5 (41.7)	7 (58.3)	25.75
Pineal region tumors	3 (0.2)	1 (33.3)	2 (66.7)	52.67
Embryonal tumors	45 (3.7)	11 (24.4)	34 (75.6)	13.18
Cranial and paraspinal nerve tumors	57 (4.7)	28 (49.1)	29 (50.9)	46.40
Meningiomas	290 (24.1)	216 (74.5)	74 (25.5)	55.78
Mesenchymal tumors	21 (1.7)	8 (38.1)	13 (61.9)	35.14
Lymphomas	14 (1.2)	8 (57.1)	6 (42.9)	53.07
Germ cell tumors	44 (3.7)	19 (43.2)	25 (56.8)	29.36
Sellar region tumors	72 (6)	37 (51.4)	35 (48.6)	43.11
Metastatic tumors	256 (21.3)	78 (30.5)	178 (69.5)	56.12
Total	1,204 (100)	567 (47.1)	637 (52.9)	48.82

Among CNS nervous system metastases, lung tumors were seen in 58%, breast tumors in 16%, tumors of unknown primary origin (TUP) in 5%, colon tumors in 4%, gynecologic tract tumors in 3.1%, and kidney, stomach, and bladder tumors in 2% equally. Of those with lung tumors, 89.2% were male and 10.8% female. In all cases, 69.5% were located in the cerebrum, 28.1% in the cerebellum, and 2.3% in the spinal cord. Of the lung metastases, 58.8% were adenocarcinoma, 21.6% were squamous cell carcinoma, 15.5% were neuroendocrine carcinoma (NEC), and 4.1% were other tumors. Of the breast carcinomas, 60.1% consisted of invasive ductal carcinoma and 39% of other tumors. There was one male case among breast metastases. The primary origin, histological type, gender, and localization distribution of the patients are summarized in Table 2.

**Table 2:** Primary origin, histological type, gender, and localization characteristics of metastatic central nervous system tumors SCC: squamous cell carcinoma

Primary origin and histological type	n (%)	Female (n(%))	Male (n(%))	Cerebrum (n(%))	Cerebellum (n(%))	Spinal (n(%))
Lung	148 (58)	16 (10.8)	132 (89.2)	101 (68.2)	46 (31.1)	1 (0.7)
Adenocarcinoma	87 (58.8)					
SCC	32 (21.6)					
Neuroendocrine carcinoma	23 (15.5)					
Other	6 (4.1)					
Breast	41 (16)	40 (97.6)	1 (2.4)	28 (68.3)	12 (29.3)	1 (2.4)
Invasive ductal carcinoma	25 (61)					
Other	20 (39)					
Tumors of unknown primary origin	13 (5)	5 (38.5)	8 (61.5)	6 (46.1)	5 (38.5)	2 (15.4)
Neuroendocrine carcinoma	5 (38.4)					
Poorly differentiated carcinoma	5 (38.4)					
SCC	2 (15.3)					
Malignant melanoma	1 (8)					
Colon (adenocarcinoma)	10 (4)	5 (50)	5 (20)	8 (80)	2 (20)	
Kidney (clear cell carcinoma)	5 (2)		5 (100)	3 (60)	2 (40)	
Gynecologic tract	8 (3.1)	8 (100)		7 (87.5)	1 (12.5)	
Serous carcinoma (ovary)	4 (50)					
Clear cell carcinoma (ovary)	1 (12.5)					
SCC (cervix)	2 (25)					
Endometrioid carcinoma (uterus)	1 (12.5)					
Stomach (adenocarcinoma)	5 (2)	1 (20)	4 (80)	3 (60)	1 (20)	1 (20)
Bladder	5 (2)		5 (100)	4 (80)	1 (20)	
Skin (malignant melanoma)	4 (1.6)		4 (100)	4 (100)		
Adrenal (neuroblastoma)	4 (1.6)		4 (100)	4 (100)		
Bone	2 (0.8)		2 (100)	2 (100)		
Nasal cavity	2 (0.8)	1 (50)	1 (50)	2 (100)		
Soft tissue	2 (0.8)	1 (50)	1 (50)	2 (100)		
Prostate	2 (0.8)		2 (100)	1 (50)	1 (50)	
Esophagus	2 (0.8)	1 (50)	1 (50)	2 (100)		
Liver	1 (0.4)		1 (100)	1 (100)		
Larynx	1 (0.4)		1 (100)		1 (100)	
Testis	1 (0.4)		1 (100)			1 (100)
Total (n(%))	256 (100)	78 (30.5)	178 (69.5)	178 (69.5)	72 (28.1)	6 (2.3)

In TUP, the diagnosis of neuroendocrine carcinoma was made with cytokeratin and synaptophysin positivity in tumors with histologically neuroendocrine features. Histologically, tumors consisting of cells with large cytoplasm, hyperchromatic pleomorphic nuclei, and solid growth patterns without glandular morphology were diagnosed as metastatic carcinoma (poorly differentiated carcinoma) with cytokeratin positivity. p63-positive tumors with epithelial morphology were diagnosed as squamous cell carcinoma. Melan-A-positive tumors with or without melanin pigmentation, consisting of infiltration of cells with epithelioid/spindle-shaped, hyperchromatic, pleomorphic nuclei and large eosinophilic nucleoli, were diagnosed as malignant melanoma. The immunohistochemical panel and staining results applied in tumors of unknown primary origin are summarized in Table 3.

**Table 3:** Immunohistochemical features of tumors of unknown primary origin NEC: neuroendocrine carcinoma; PDC: poorly differentiated carcinoma; SCC: squamous cell carcinoma; MM: malignant melanoma; GFAP: glial fibrillary acidic protein; PanCK: pan-cytokeratin; CK7: cytokeratin 7; CK20: cytokeratin 20; TTF-1: thyroid transcription factor 1; Syn: synaptophysin; Chr: chromogranin; LCA: leukocyte common antigen; CD56: cluster of differentiation 56; CDX2: caudal type homeobox transcription factor 2; Melan-A: melanoma antigen; ER: estrogen receptor Immunohistochemically positive staining is indicated by "+," negative staining by "-," focal positivity by "F(+)," and markers not applied for that case by "N."

	GFAP	PanCK	CK7	CK20	TTF-1	Syn	Chr	LCA	CD56	CDX2	Melan-A	p63	p40	ER
NEC	-	+	+	-	+	+	+	-	N	N	N	N	N	N
NEC	-	+	+	-	N	+	-	N	+	-	-	N	N	N
NEC	-	+	+	-	N	+	+	-	N	N	N	N	N	N
NEC	-	N	N	N	+	+	+	N	N	N	N	-	-	N
NEC	-	+	N	N	+	+	+	N	N	N	N	+	N	N
PDC	-	+	+	F(+)	-	-	-	N	N	F(+)	-	-	N	N
PDC	-	F(+)	-	-	-	-	N	N	N	F(+)	-	-	N	N
PDC	-	+	-	-	-	-	-	-	N	-	-	-	N	N
PDC	-	N	+	-	-	N	N	N	N	N	N	-	N	-
PDC	-	+	+	-	-	-	-	N	N	-	-	-	N	-
SCC	-	+	N	N	-	N	N	N	N	N	N	+	N	N
SCC	-	+	-	N	N	N	N	N	N	N	N	N	+	N
MM	-	-	-	-	-	N	N	N	N	N	+	N	N	N

## Discussion

CNS metastases are the most common intracranial malignancies in adults, and brain metastases were found in 25% of patients who died of cancer in autopsy studies. In the USA, 170,000 new cases are reported annually [2,7]. According to the WHO, confirmed or unconfirmed primary CNS tumors constitute 85%-90% of all brain tumors, while metastatic tumors are seen in approximately 10% [1]. In addition, the incidence of intracranial metastases in various epidemiological studies varies between 2.8 and 11.1 per 100,000 people [8-10]. CNS metastases are seen 80% in the cerebral hemispheres, 15% in the cerebellum, and 5% in other areas of the CNS. CNS metastases, which mostly manifest with symptoms of increased intracranial pressure in the clinic, may manifest as intracranial hemorrhage and infarction areas that can be easily recognized by MRI and CT in some patients [1]. MRI, one of the diagnostic methods, has high specificity and sensitivity in these patients [2,11-13]. Most of the patients primarily referred to the neurology or neurosurgery are due to neurological symptoms [14]. The most common complaints at presentation are neurological deficits, seizures, and headaches, while few patients were asymptomatic. The reasons for these complaints are mass effect, cerebral edema, and increased intracranial pressure [15]. Treatment options include surgery, radiotherapy, and chemotherapy within the clinical indications of the patients, as well as antiepileptics and corticosteroids [16]. It has been reported that there is an increase in survival with combined treatments applied over several decades in patients with CNS metastases [17-19]. The main criteria determining the prognosis in patients with CNS metastases are patient age, Karnofsky performance status, number of brain metastases, and presence of extracranial disease [1]. Other factors of prognostic significance are the specific tumor type and the molecular markers involved (e.g., CerbB2 in breast cancer) [1]. While it has been reported in different studies that the most common intracranial mass lesion is metastatic tumors [2,20-22], in our series, when we grouped them according to the WHO 2016 classification, metastatic tumors, either only intracranial or within all CNS masses, were the third most common after astrocytic and oligodendral tumors and meningiomas. However, similar to our study, there are also series reporting that metastases are at a lower rate than primary lesions among all CNS malignancies [3,23]. While brain metastases are caused by GIS, prostate, and lung tumors in men, it is caused by breast, lung, GIS, and other system tumors in women. Likewise, the most common histological type varies according to the age of the patient [1,3]. The mean age was higher than that of primary CNS tumors [23,24]. In our series, metastatic CNS tumors were more common in males. Although 19.1% of our cases were breast and gynecological tumors and only 1.2% were prostate and testicular tumors, when all metastatic lesions were evaluated together, the male/female ratio was 2.28, while in other studies, it was 2.3 and 1.2 [23,24]. The histological features of CNS metastases can vary as much as their primary origin. Lung malignancies were the most common metastatic CNS tumors. While this rate ranged between 12% and 65% in studies, this rate was 58% in our series, which was higher than that in the other two studies with a higher number of cases [21]. In these studies, it was found to be 34% and 35.6%. Histological diagnosis was not emphasized in most series evaluating data on CNS metastases. Only a few studies have reported data on this. Although detailed information in terms of histological diagnosis was not provided in these studies, the most common histological diagnosis was found to be adenocarcinoma, both in all central nervous system metastases and especially in lung metastases. Our study supported these findings, and adenocarcinomas (Figure 1) were followed by squamous cell carcinomas and neuroendocrine carcinomas among lung metastases [23,25,26]. Breast tumors were the most common in women (Figure 1).

**Figure 1:** Lung and breast metastases A: Lung adenocarcinoma metastasis exhibiting papillary and micropapillary morphology with adjacent inflamed glial tissue (hematoxylin and eosin: 100×). B: Immunohistochemical stain TTF-1 showing nuclear positivity in the tumor cells (100×). C: Metastatic breast carcinoma no special type (NST) infiltrating the glial tissue (hematoxylin and eosin: 100×). D: Immunohistochemical stain GATA3 showing nuclear positivity in the tumor cells (100×).

This was followed by lung, TUP, gynecologic tract, and colon tumors. Invasive carcinoma no special type (NST) was the most common diagnosis among breast tumors. Lung, TUP, colon, kidney, bladder, stomach, and skin (malignant melanoma) tumors were most common in men. In a study of a 20-year series, the most common tumors seen in men were lung (44%), followed by malignant melanoma (12%), colorectal (9%), and prostate (9%). In women, lung and breast tumors were found at an equal rate (33%) [27]. When we compare our data, it can be said that these different rates arise from regional differences because, in studies from different regions, breast metastases were the second most common after lung in all adults [10,23]. In our series, TUP were seen in the third frequency after lung and breast tumors. Among these tumors, neuroendocrine carcinomas (Figure 2) and poorly differentiated carcinomas were seen with equal frequency (38.4). This rate was found to be higher in other studies (14%) [28].

**Figure 2:** Neuroendocrine carcinoma metastasis A: Infiltration of cells with pleomorphic vesicular nuclei and granular cytoplasm (hematoxylin and eosin: 100×). B. Immunohistochemical stain chromogranin showing paranuclear Golgi-like cytoplasmic positivity in the tumor cells (100×).

While gynecologic tract tumors were seen at a rate of 3.1% in our study, this rate was 6.6% and 5.6%, respectively, in other similar studies, which is higher than our study [27,28]. Among these tumors, ovarian serous carcinomas are the most common. All of this patient group had been diagnosed previously. In our study, unlike similar studies, malignant melanoma and prostate carcinoma metastases were observed rarely [27]. The immunohistochemical markers frequently used in CNS metastases (CK5/6, CD56, CK7, CK20, TTF-1, napsin A, GCDFP-15, CDX2, RCC, PSA, EMA, PAX8, vimentin, and Melan-A) are very useful for the diagnosis of the primary tumor [6]. In our cases, cytokeratin 7, TTF-1, p63, and p40 for lung tumors; CK7, GATA3, and GCDFP-15 for breast tumors; and cytokeratins, synaptophysin, chromogranin, and CD56 for neuroendocrine tumors were the most used markers. In addition to clinical history, radiological findings, and histomorphology, the primary diagnosis was mostly reached with immunohistochemical panels containing these markers. Since the patient group without clinical history and radiological primary tumor is the third largest group of central nervous system metastases, the pathological evaluation and immunohistochemical markers to be applied in these patients are even more important.

Among the tumors of unknown primary origin, neuroendocrine carcinoma, squamous cell carcinoma, and malignant melanoma metastasis were diagnosed in our cases. Although the immunohistochemical panel applied after morphological evaluation in CNS metastatic tumors in our center varies between pathologists, different immunohistochemical stains were applied to determine the histological origin and primary origin of the tumor. Cytokeratin, GFAP, and TTF-1 have generally been applied in addition to synaptophysin and chromogranin in NECs. In addition to this panel, Melan-A, CDX2, p63, or p40 were added to patients diagnosed with poorly differentiated carcinoma metastasis. Cases with squamous cell carcinoma were diagnosed with TTF-1 negativity and positive expression of p63 and p40.

The limitations of our study are that the cases included in the tumor group of unknown primary origin in our department were based on our hospital’s information system and that different immunohistochemical panels were used among different pathologists in the approach to these tumors, and molecular study was not done.

## Conclusions

The most common metastatic tumors in the CNS are lung metastases in men and breast carcinoma metastases in women, and our findings include various differences from the literature in terms of frequency and ratio. It is possible to make a diagnosis with a more limited immunohistochemical panel in patients with a history of lung or breast malignancy or known to have a lung mass. However, it should not be forgotten that a primary tumor origin may not be found in a significant group. Neuroendocrine tumors and poorly differentiated carcinoma constitute most of this group. Therefore, in routine pathology practice, the task of the pathologist should be to first try to collect data about the differential diagnosis of the metastatic tumor after distinguishing it from the primary CNS tumors. Unnecessary immunohistochemical staining should be avoided because it will increase both the workload and the cost.
